The article "Risk Factors for Venous Thrombosis after Spinal Surgery: A Systematic Review and Meta-analysis" was published in 2022. Journal: Comput Math Methods Med.

# Risk Factors for Venous Thrombosis after Spinal Surgery: A Systematic Review and Meta-analysis

**DOI:** 10.1155/2022/1621106

**Published:** 2022-03-27

**Authors:** Sheng Wang, Leilei Wu

**Affiliations:** Affiliated Hospital of Weifang Medical University, Spine Surgery, 261031 Weifang, Shandong, China

## Abstract

**Background:**

Venous thrombosis, comprising DVT and PE, is an orthopedic condition that may be fatal after surgery. This study's purpose was to analyze risk factors for venous thrombosis following spine surgery to help guide treatment prophylaxis.

**Methods:**

A computer searched English databases such as PubMed, Web of Science, Embase, Cochrane Library, and Google Academic for relevant publications after spinal surgery. Preoperative walking difficulties, hypertension, diabetes, heart disease, preoperative bleeding volume, etc., were all examined using the NOS scale. Data were analyzed using Review Manager 5.3 software. An analysis was done. Due to the study's differences, the data was compiled using fixed effects or random effects models.

**Results:**

A total of 25 studies were considered, with a total of 1,927,781 individuals after spine surgery, including 7843 patients with venous thrombosis. The included literatures had NOS scores ranging from 5 to 8. According to the findings of the meta-analysis, the age of patients with venous thrombosis after spinal surgery (OR = 7.53, 95% CI (6.73, 8.33)), blood loss (OR = −141.79, 95% CI (-154.68, -128.9), *P* = 0.00001), and operation time (OR = 76.93, 95% CI (73.17, 80.86), *P* = 0.00001) were higher than those without; diabetes mellitus (OR =1.23, 95% CI (1.12, 1.34), *P* = 0.00001) and walking disability history (OR = 2.97, 95% CL (1.77, 4.98), *P* = 0.0001) increased the incidence of postoperative venous thrombosis.

**Conclusion:**

High age, female, spinal fusion, big volume blood loss patients, operation time, and hypertension, diabetes, and walking issue are all risk factors for venous thrombosis following surgery.

## 1. Introduction

Patients having major orthopedic surgery (DVT) have an increased risk of venous thromboembolism, which may include pulmonary embolism (PE) and deep venous thrombosis [1]. VTE is a well-known and feared surgical complication, as well as a leading cause of death [2]. Acute thromboembolic illness (VTE) may result in substantial morbidity, poor quality of life, and even death [3]. It may also lead to increased medical costs and a considerable financial burden on individuals and their families [4]. The use of pharmacological prophylaxis is well established in a variety of surgical procedures, most notably hip and knee replacements, for which there are well-established criteria and dosing guidelines [5]. Chemoprophylaxis recommendations in spinal surgery are less well defined, and there are currently no clear evidence-based standards in this discipline [6]. Because there is no consensus on the efficacy and safety of chemoprophylaxis in spine surgery, a wide range of treatment options are available, many of which are dependent on the surgeon's personal experiences with the medication [7]. As a consequence, spine surgeons must be aware of the prevalence of VTE as well as the risk factors that contribute to the development of this condition [8].

The article "Risk Factors for Venous Thrombosis after Spinal Surgery: A Systematic Review and Meta-analysis" was published in 2022. Journal: Comput Math Methods Med.

An epidural hematoma, a devastating but rare complication of spinal surgery, may occur from bleeding issues [9]. As a consequence, spine surgeons should use caution when prescribing anticoagulants. To balance VTE morbidity and mortality with epidural hematomas' potential of permanent neurological disability, they must decide [10]. Many researchers have looked at the VTE risk factors following spine surgery [11]. Due to the limited sample sizes and varying detection technology, the incidence varies [12]. These studies found that older patients on prolonged bed rest for paralysis or pain had a higher incidence of VTE than younger patients [13]. Although variables such as the presence or absence of D-dimer in the blood [14], the length of the operation, intraoperative blood loss, and surgical procedures all have an effect on the frequency of VTE after spine surgery, the incidence remains consistent and never paradoxical [15].

A comprehensive review of the available literature was conducted in order to get a better understanding of VTE incidence and risk factors in patients undergoing spine surgery. In order to assist surgeons in making well-informed therapy choices, evidence-based information about this subject will be presented in a straightforward way.

## 2. Materials and Methods

### 2.1. Search Strategy

Search the computer for PubMed, Web of Science, Embase, Cochrane Library, and other English databases. The English search terms are “Spinal surgery”, “Venous thrombosis”, and “spine”, all from the medical topic word list (mesh). The retrieval term for all databases is from the time the database was created until December 30, 2021. In addition, in order to completely include the literature, several references were manually gathered.

### 2.2. Inclusion and Exclusion Criteria

All of the studies that were included were studies that were based on what people saw and did on the incidence of venous thrombosis after spine surgery. The following factors are included: (1) age, (2) gender, (3) BMI, (4) history of hypertension, (5) diabetes history, (6) history of heart disease, (7) preoperative D-dimer level, (8) history of preoperative walking problem, (9) mode of surgery, (10) mode of anesthesia, (11) surgical location, (12) duration of operation, (13) blood loss, (14) smoking history, (15) alcohol history, and (16) postoperative infection. At least one of the aforementioned signs may be found in the included literature. Criteria for exclusion include (1) a summary study, (2) an expert opinion, (3) a case report or case series report, (4) preoperative or coagulation function abnormal and clinically significant, (5) venous thrombosis occurred before the procedure, (6) blood system illnesses, (7) various thrombus prevention techniques were utilized both before and after the operation, and (8) after contacting the author, the relevant information could not be obtained.

The article "Risk Factors for Venous Thrombosis after Spinal Surgery: A Systematic Review and Meta-analysis" was published in 2022. Journal: Comput Math Methods Med.

### 2.3. Selection of Studies

Two investigators independently reviewed all of the subjects, abstracts, and full texts of the literature that had been chosen. Following that, the eligible studies were selected in accordance with the inclusion criteria. Discussion and consensus were used to address any disagreements that arose among the investigators. A third author was sought to help settle the situation when no agreement could be obtained.

### 2.4. Data Extraction and Quality Assessment

Two researchers independently extracted the data, which included the name of the original author, the year of publication, the country of origin of the subjects, and information on numerous inclusion indicators indicated in the inclusion criteria. If there are disagreements, they must be handled by conversation; if the dispute cannot be resolved, the third researcher must be consulted. Two researchers extracted the data independently, including the first author's name, the year of publication, the country of the study population, and the details on numerous inclusion indicators indicated in the inclusion criteria. If there are disagreements, they must be handled by conversation; if the dispute cannot be resolved, the third researcher must be consulted.

### 2.5. Statistical Analysis

For meta-analysis, Review Manager 5.3 software was employed. The analysis statistics were odds ratio (OR) or relative risk (RR); the measurement data analysis statistics were weighted mean difference (WMD) or standardized mean difference (SMD), and each effect quantity was given by a 95% confidence interval (95% CI). The *Q* test and *I*^2^ were used to quantify the heterogeneity of the research. When *P* > 0.1 and *I*^2^ > 50%, it is assumed that the heterogeneity is not significant, and the fixed effect model is used to combine the data. When *P* < 0.1, which is 50%, it is assumed that the heterogeneity is substantial, and the fixed effect model is used to integrate the data. The model with a random effect is used, and the cause of heterogeneity is identified as thoroughly as feasible for subgroup analysis. If the reason for heterogeneity cannot be determined, the random effect model is utilized in meta-analysis. There was a statistically significant difference between the two groups (*P* < 0.05).

The article "Risk Factors for Venous Thrombosis after Spinal Surgery: A Systematic Review and Meta-analysis" was published in 2022. Journal: Comput Math Methods Med.

## 3. Results

### 3.1. Selected Study Results

The approach for screening and selecting articles for inclusion in this study is shown in Figure 1. Initially, a total of 2139 studies were discovered. 491 were eliminated for duplicate entries, and 1600 were excluded following a title/abstract assessment. The remaining 48 papers were then subjected to a full-text review. 23 of them were rejected because they did not match the qualifying requirements. Finally, 25 papers satisfied the inclusion criteria and were included in our meta-analysis; the features of these studies are shown in Table 1. One of the 25 studies was meant to be prospective, while the other 24 were planned to be retrospective. The entire number of participants in the study was 3,215,173, of which 1038 were difficult to deal with VTE, and the overall occurrence of VTE following spine surgery was 0.35% (the original studies' occurrence of VTE was 0.15–29.38%). VTE occurred in 8.43% of patients from Asians and 0.33% of Western patients; the difference is statistically significant (*P* < 0.0001).

### 3.2. Data Quality Assessment

All 14 studies were critically appraised independently by the two reviewers. The study design and outcome measure were valid and appropriate to the research questions. The risk of bias in the study design and results was assessed by the revised Cochrane risk of bias in randomized trials (RoB 2) latest version 22 August 2019 (Figure 2).

### 3.3. Risk Factor Summary

#### 3.3.1. Age Factor

A total of 8 studies including 6629 people [11–18, 35], including 459 cases of VTE (+) and 6170 cases of VTE (-), discovered a connection between age and the risk of venous thrombosis after spine surgery. The random effect model was used for meta-analysis since the studies displayed statistical heterogeneity (*I*^2^ = 70%, *P* = 0.001). The results showed that the mean age of VTE (+) patients following spinal surgery was older than that of VTE (-), and the difference was statistically significant (OR = 7.53, 95% CI (6.73, 8.33)) (Figure 3), *P* < 0.00001.

#### 3.3.2. Gender Factor

Nine studies comprising 10,500 patients found a link between gender and the incidence of venous thrombosis following spine surgery [15–23, 35], with 256 instances of VTE (+), 282 cases of VTE (-), 5235 men, and 5265 females. Because the studies had statistical heterogeneity (*F* = 70%, *P* = 0.0005), the random effect model was employed for meta-analysis. Incidence of venous thrombosis following spinal surgery in female or male patients has no significant difference (OR = 0.77, 95% CI (0.64, 0.93), *P* = 0.06, Figure 4).

The article "Risk Factors for Venous Thrombosis after Spinal Surgery: A Systematic Review and Meta-analysis" was published in 2022. Journal: Comput Math Methods Med.

#### 3.3.3. BMI

Five studies [16–20, 35] found a link between BMI and postoperative venous thrombosis. There are two for Chinese and two for foreigners. In the study sample, there were 378 instances of VTE (+) and 5196 cases of VTE (-). Because the studies had considerable statistical heterogeneity (*I*^2^ = 87 percent, *P*0.00001), the random effect model was employed for meta-analysis. Those with VTE (+) had a lower mean BMI than patients with VTE (-) (Figure 5).

#### 3.3.4. Operation Methods

Six studies comprising 49,389 patients found an association between surgical procedures and the prevalence of venous thrombosis following spine surgery, including 32,032 patients with nonfusion and 17,357 patients without fusion [23–29]. Because there was no significant heterogeneity across the studies, the model with a fixed effect was adopted for meta-analysis. The findings revealed that the frequency of VTE in patients with nonfusion was greater than that in patients with fusion. There was a statistically significant difference between the two (OR = 1.67, 95% CI (1.40, 1.99), *P* = 0.00001, Figure 6).

#### 3.3.5. Operative Approach

Three studies comprising 461 patients found a relationship between surgical approach and the frequency of venous thrombosis following spine surgery [21–23], including 328 instances of posterior surgery, 133 cases of anterior/posterior mixed surgery, 34 cases of VTE (+), and 427 cases of VTE (-). The fixed effect model was adopted for meta-analysis since there was no statistical heterogeneity across the studies. The data revealed that the incidence of VTE was higher in patients undergoing simple posterior surgery than in patients undergoing anterior/posterior combination surgery, although the difference was not statistically significant (OR = 0.63, 95% CI (0.32, 1.25), *P* = 0.30, Figure 7).

#### 3.3.6. Operative Site

Four investigations including 1617 patients found a link between the surgical site and the incidence of venous thrombosis following spinal surgery [12–16], including 285 instances of cervical surgery, 1332 cases of thoracolumbar surgery, 75 instances of VTE (+), and 1542 instances of VTE (-), because there was no statistically significant difference between the studies (*I*^2^ = 0, *P* = 0.59). In this meta-analysis, the fixed effect model was used as a basis. The findings revealed that the incidence of VTE was lower in cervical surgery patients than in thoracolumbar surgery patients (OR = 1.17, 95% CI (0.66, 2.08), *P* = 0.59, Figure 8).

The article "Risk Factors for Venous Thrombosis after Spinal Surgery: A Systematic Review and Meta-analysis" was published in 2022. Journal: Comput Math Methods Med.

#### 3.3.7. Duration of Surgery

A total of 8 investigations comprising 46,840 patients, including 680 instances of VTE (+) and 46,160 cases of VTE (-) [12–19, 35], indicated that the length of surgery was associated with the incidence of venous thrombosis following spine surgery. Because there was statistical heterogeneity in each research question (*I*^2^ = 98%, *P* = 0.00001), the random effect model was utilized for meta-analysis. The findings of the study revealed that the mean operation time of VTE (+) patients following spinal surgery was greater than that of VTE (-), and the difference was statistically significant (OR = 76.93, 95% CI (73.17, 80.86), *P* = 0.00001, Figure 9).

#### 3.3.8. Intraoperative Blood Loss

A total of 7 investigations comprising 3195 individuals [18–24, 35], including 256 instances of VTE (+) and 2939 cases of VTE (-), found a link between blood loss and the risk of blood clots following spine surgery. Because there was statistical heterogeneity in each trial (*I*^2^ = 100%, *P* = 0.00001), the random effect model was utilized for meta-analysis. Because of the considerable differences in mean blood loss across trials, SMD was utilized as the statistic. The findings of the research revealed that the mean blood loss in VTE (+) patients following spinal surgery was greater than that in VTE (-). There was a statistically significant difference between the two (OR = −141.79, 95% CI (-154.68, -128.9), *P* = 0.00001, Figure 10).

#### 3.3.9. Hypertension

Five studies including 44,306 patients found a link between hypertension and the occurrence of venous thrombosis following spinal surgery, including 20,612 patients with hypertension, 23,694 patients with no hypertension, 859 patients with VTE (+), and 43,447 patients with VTE (-) [14–18, 35]. In this meta-analysis, the fixed effect model was used since there was no substantial heterogeneity across the studies (*I*^2^ = 50%, *P* = 0.09) (Figure 11).

#### 3.3.10. Diabetes Mellitus

A total of 10 studies reported the correlation between diabetes and the incidence of venous thrombosis after spinal surgery [15–24, 35]. There were 48,676 cases involving diabetes, 90,114 cases involving nondiabetes, 2902 cases of VTE (+), and 135,888 cases of VTE (-). The research questions did not have statistical heterogeneity (*I*^2^ = 94%, *P* = 0.00001). As a result, the fixed effect model was used in the meta-analysis. Comparing diabetic individuals to nondiabetic patients, the risk of VTE increased following spine surgery.(OR = 1.23, 95% CI (1.12, 1.34), *P* = 0.00001, Figure 12).

The article "Risk Factors for Venous Thrombosis after Spinal Surgery: A Systematic Review and Meta-analysis" was published in 2022. Journal: Comput Math Methods Med.

#### 3.3.11. Heart Disease

Heart disease has been linked to a higher risk of postsurgical blood clots in four studies [20–24], involving 5718 patients, including 1550 cases of heart disease, 4168 cases of nonheart disease, 453 cases of VTE (+), and 5265 cases of VTE (-), which were not available due to statistical heterogeneity (*P* = 0.95). As a result, for the meta-analysis, a fixed effect model was adopted. The findings revealed that the incidence of VTE following spinal surgery was greater in patients with nonheart disease than in patients with heart disease; the difference was statistically significant (OR = 0.96, 95% CI (0.78, 1.20), *P* = 0.74, Figure 13).

#### 3.3.12. Preoperative D-Dimer

Six studies comprising 2994 individuals [28–33, 36], including 223 instances of VTE (+) and 2771 cases of VTE (-), found a link between preoperative D-dimer level and the instance of VTE following spinal surgery. Because the studies had statistical heterogeneity (*I*^2^ = 90%, *P* = 0.00001), the random effect model was employed for meta-analysis. The findings revealed that the mean preoperative D-dimer level in VTE (+) patients following spinal surgery was greater than that in VTE (-) (OR = −0.08, 95% CI (-0.14, -0.01), *P* = 0.02, Figure 14).

#### 3.3.13. Preoperative Walking Dysfunction

Five investigations comprising 1671 patients found a link between preoperative walking dysfunction and the occurrence of VTE following spine surgery [30–33, 36], with 82 patients having walking dysfunction, 1589 having no walking dysfunction, 168 having VTE (+), and 1503 having VTE (-). Since there was no statistical heterogeneity across the studies, the fixed effect model was used in the meta-analysis. The findings revealed that individuals with preoperative nonwalking dysfunction had a greater incidence of VTE following spine surgery than those with walking impairment. There was a substantial statistical difference (OR = 2.97, 95% CL (1.77, 4.98), *P* = 0.0001, Figure 15).

#### 3.3.14. Publication Bias

Begg and Egger tests revealed no evidence of publication bias in any of the papers included in this review (Figure 16).

## 4. Discussion

Complications from spine surgery cause people bodily, emotional, and social distress. These two incidents have diminished the surgical result and worried spinal surgeons. A deep epidural hematoma may compress the spinal nerve root, causing substantial neurological issues, and a severe venous embolism can swiftly kill the patients [34]. Although medications may effectively prevent venous thrombosis, the risk of venous thrombosis following spine surgery is significantly smaller than after joint surgery [37]. However, several investigations have demonstrated that deadly PE has much more severe repercussions and medical risks than epidural hematoma [38]. If surgical patients' venous thrombosis prevention and treatment are ignored, preventable PE will endanger the patient's life. Indicator measurement is difficult due to various aspects such as research design, sample size, and subject inclusion/exclusion criteria [39]. The incidence of venous thrombosis following spinal surgery varies between 0.31% and 31%, showing that there is no unanimity on the occurrence. Moreover, the existing system assessment findings vary. So, through meta-analysis/systematic review, in line with the inclusion and exclusion criteria, a more extensive qualitative and quantitative synthesis of previous research is required to investigate the risk factors for thrombosis following spine surgery.

The article "Risk Factors for Venous Thrombosis after Spinal Surgery: A Systematic Review and Meta-analysis" was published in 2022. Journal: Comput Math Methods Med.

In terms of surgery, fusion vs. nonfusion, blood loss (big), operation duration (long), past history face, hypertension (+), diabetes (+), preoperative walking problem (+), and thrombosis risk following spinal surgery [40], thrombosis in spinal surgery is linked to the following variables, with close correlation to (1) trauma, blood loss, and blood transfusion caused by operation damaging intima of blood vessels and making the body hypercoagulable; (2) compression of the venous system caused by long-lying posture during operation, such as inferior vena cava, iliac vein, and femoral vein; (3) implantation of metal and other artificial materials, such as pedicle screw system, bone cement, and artificial bone; (4) anesthesia, especially general anesthesia; (5) lower limb paralysis occurrence. Lower limbs lose muscular pump and vasomotor reflex function; (6) changes in body fluid balance, electrolyte imbalance, and fluctuation of the internal environment during the perioperative period; and (7) staying in bed or break for a long time after surgery. These are connected to the three pathogenic components of venous thrombosis: vascular wall damage, sluggish blood flow, and hypercoagulable condition. The beginning of any factor may result in thrombosis. A high quantity of glucose in the blood might cause blood. Meta-analysis research found that vascular endothelial damage increased the risk of blood coagulation (OR = 1.49, 95% CI (1.40, 1.58), *P* = 0.00011); the result of this research is comparable [41].

Studies on the occurrence of venous thrombosis after column surgery have been reported; however, the results are mixed [42]. Compare this study's results to prior studies' findings on hypertension (+), diabetes (+), preoperative walking difficulty (+),surgery (fusion), age, gender, blood loss, and operation time (long). This study found a statistically significant difference in the incidence of venous thrombosis after spine surgery due to these variables [43]. This is because, in terms of age-related venous thrombosis incidence, this investigation included five previously published studies that complimented the results and increased the sample size. The data suggest that age may be a risk factor for postsurgery thrombosis. In terms of gender and venous thrombosis incidence, this study excluded case-control studies (the researchers believe the control selection is not representative) and studies utilizing prophylactic methods in favor of three newly published studies [44]. Gender may be a risk factor for thrombosis following spine surgery. However, it is unclear if gender (for example, men) is a risk or protective factor for thrombosis. Based on Zacharia et al., this study comprised five investigations on the impact of blood loss on venous thrombosis incidence [45]. Because blood loss varies widely, SMD was used in this study. The number of fused segments and hand operation method may be linked to heterogeneity. This study included seven studies on the impact of operation time on venous thrombosis incidence, increasing sample size, and statistical accuracy. However, the included studies are quite varied, maybe related to surgical method, bleeding volume, or other factors. The patient's condition and personal will, as well as the doctor's evidence-based decision-making, impact the operation time and amount of bleeding, as well as the hemostasis caused by intraoperative bleeding.

The article "Risk Factors for Venous Thrombosis after Spinal Surgery: A Systematic Review and Meta-analysis" was published in 2022. Journal: Comput Math Methods Med.

The comparison of BMI and the incidence of venous thrombosis after spinal surgery revealed that the heterogeneity of the included studies was substantial, and the difference was not statistically significant [46]. The source of heterogeneity was investigated using subgroups of the study population. Following subgroup analysis, the heterogeneity of each subgroup fell dramatically, suggesting that the population may be the cause of the considerable heterogeneity across groups. The mean value of BMI difference in various Asian populations is demonstrated to be in the other direction. It implies that BMI may not be a direct cause of venous thrombosis following spine surgery but may have an indirect effect on the establishment of postoperative thrombosis. Intermediate elements include vascular elasticity, blood viscosity, and the degree of vascular wall damage. This research also discovered that there was no significant difference in preoperative D-dimer levels between the postoperative VTE (+) group and the VTE (-) group. It is stated that the present data are insufficient to show that the difference in preoperative D-dimer levels has a statistically significant influence on the incidence of venous thrombosis following spine surgery. Large sample size and multicenter research are required. At the same time, consider the influence of the dynamic shift in postoperative D-dimer level on thrombosis.

The article "Risk Factors for Venous Thrombosis after Spinal Surgery: A Systematic Review and Meta-analysis" was published in 2022. Journal: Comput Math Methods Med.

## 5. Limitations

Age, gender, BMI, surgery time, and blood loss were all taken into account. They propose that where there is little or no heterogeneity, analytical meta-analysis may help determine effect sizes or test hypotheses. Methodological, clinical, or statistical variables may all contribute to heterogeneity. The majority of the papers in this study are retrospective NOS score investigations. Biases exist in certain literatures, such as (1) research bias due to disparities in inquiry methods between venous and nonvenous thrombosis situations; responders and investigators may make systematic mistakes. Concern about the patient's medical history, for example, varies. (2) The study's major result and measurement bias were not addressed, and there were no consistent diagnostic criteria across trials; neither are preoperative diagnostic criteria for walking dysfunction or hypertension. Variable and method heterogeneity may be included in the meta-analysis. Oral vitamin E, pregnancy-preventive medicines, aspirin, postoperative functional activity, postoperative braking, and other factors contributed to clinical variability. These signs have not received much attention. Their absence might result in phenotypic differences. As a consequence, age and gender are exaggerated or minimized, resulting in clinical diversity. Clinical variability may emerge as a result of surgical skill, competency, and illness severity, all of which influence operation duration and blood loss. The unequal distribution of these components causes variation in study outcomes. There was insufficient data in the included trials, and there was no subgroup analysis to determine the cause of heterogeneity.

## 6. Conclusion

However, there is no strong evidence that these characteristics are independent risk factors for postoperative thrombosis. Diabetes may be caused by vascular endothelial damage, which is an indirect risk factor for venous thrombosis and poor cardiac function. Insufficient energy may restrict activities and produce lower extremity venous stasis (nonindependent risk variables). Large-scale multicenter prospective research is needed to evaluate the incidence of venous thrombosis following spine surgery. Regardless, this investigation found venous thrombosis following spine surgery. Birth-related risks need the spinal surgeon to focus on the postoperative period. Venous thrombosis is deadly for screening and surveillance of people with venous thrombosis. Concerning postoperative venous thrombosis prevention and therapy, a systematic review and meta-analysis based on high-quality original research are still required.

The article "Risk Factors for Venous Thrombosis after Spinal Surgery: A Systematic Review and Meta-analysis" was published in 2022. Journal: Comput Math Methods Med.

## Figures and Tables

**Figure 1:** Document screening process.

**Figure 2:** Document quality evaluation.

**Figure 3:** Age and incidence of venous thrombosis after spinal surgery.

**Figure 4:** Forest plot of incidence of venous thrombosis after spinal surgery.

**Figure 5:** Forest plot of body mass index and incidence of venous thrombosis after spinal surgery.

**Figure 6:** Forest chart of operative methods and incidence of venous thrombosis after spinal surgery.

**Figure 7:** Forest chart of the incidence of venous thrombosis after surgical approach and spinal surgery.

**Figure 8:** Forest plot of surgical site and incidence of venous thrombosis after spinal surgery.

**Figure 9:** Forest diagram of operation duration and incidence of venous thrombosis after spinal surgery.

**Figure 10:** Forest plot of bleeding volume and incidence of venous thrombosis after spinal surgery.

**Figure 11:** Forest plot of blood pressure and incidence of venous thrombosis after spinal surgery.

**Figure 12:** Forest chart of urinary disease and incidence of venous thrombosis after spinal surgery.

**Figure 13:** Forest chart of incidence of venous thrombosis after heart disease and spinal surgery.

**Figure 14:** Forest diagram of D-dimer level and incidence of venous thrombosis after spinal surgery.

**Figure 15:** Forest diagram of preoperative walking disorder and the incidence of venous thrombosis after spinal surgery.

**Figure 16:** Publication bias funnel plot.

**Table 1:** Characteristics of included research literature.

Study	Participant	Methods	Conclusion
Ikeda T [11]	194	Postoperative DVT	Perioperative application of DUS for detecting DVT in the lower extremities should be performed on patients undergoing spine surgery who are female, nonambulatory, and with higher preoperative D-dimer serum level
Boonyawat K [12]	200	Literature search	In clinical practice, the rate of VTE prophylaxis varies and may be inadequate in some centers
Park JH [13]	21,261	Generated by extracting patients with disease codes of spine surgery and VTE from the Health Insurance Review & Assessment Service National Inpatient Sample in 2014	On the basis of the incidence of VTE and the risk factors, more active prophylaxis is suggested for patients in the Korean population who undergo spine surgery
Wei J [14]	2861	Diagnosis of preoperative deep vein thrombosis (DVT) was confirmed by Doppler ultrasonography	Age, positive preoperative plasma D-dimer level, and rheumatoid arthritis had an influential impact on the incidence of DVT admitted for PLIF
Yoshioka K [15]	459	Investigated the occurrence of VTE after degenerative spinal surgery	The prevalence of VTE after elective spinal surgery was different in each group
Liu JM [16]	2715	Patients who underwent posterior lumbar spinal decompression surgery between January 2010 and August 2016 were included in this study, and their medical records were retrospectively reviewed	Blood type A, increased estimated blood loss, and prolonged surgical duration were identified as the independent risk factors for postoperative SEH with two new risk factors
Dhillon ES [17]	6869	Retrospectively examined records from 6869 consecutive spinal surgeries performed in their departments at Northwestern University	Administering anticoagulation therapy from 1 day before to 3 days after surgery is safe for patients at high risk for VTE
Akeda K [18]	737	ASD patients with VTE were identified in a prospective, multicenter database. Complications, revision, and mortality rate were examined	The incidence of VTE in ASD is 4.3% with a DVT rate of 1.9% and PE rate of 2.4%. Osteoporosis, lack of physical labor, and increased SVA correction were independent predictors of VTE
Ferree BA [19]	209	A pneumatic sequential compression device and standard compression stockings were used for primary VTE prophylaxis	DVT assessment using ultrasonography is important for proper management of VTE during the perioperative period of spinal surgery, especially for high-risk patients, such as those with advanced age or neurological deficit
Hohl JB [20]	1121	Preoperative and postoperative compression ultrasonography of the lower extremities to detect acute deep venous thrombosis (DVT)	There were no statistically significant differences in DVT rates when compared by sex, addition of one- or two-level fusion, length of procedure, or number of days of bed rest
Piper K [21]	5766	Symptomatic pulmonary emboli (PE) were diagnosed by spiral chest CT scans, nuclear scintigraphic ventilation-perfusion, and angiography	Patients with increasingly extensive surgery had a higher risk of PE, specifically those undergoing fusion of ≥5 segments
Nourian AA [22]	22,434	The American College of Surgeons National Surgical Quality Improvement Project database for the years 2006-2010 was reviewed for patients who had undergone spinal surgery according to their primary current procedural terminology code(s)	A risk score based on race, preoperative comorbidities, and operative characteristics of patients undergoing spinal surgery predicts the postoperative VTE rate. Many of these risks can be identified before surgery
Gould MK [23]	204	This retrospective review of prospectively collected data from our spine database identified 204 patients who had undergone single level (*n* = 142) or multilevel (*n* = 62) ALIF from 2008 to 2013 with minimum 6-month follow-up	Performing ALIF in the setting of spondylolisthesis or transitional anatomy resulted in higher blood loss
McLynn RP [24]	431	American College of Chest Physicians Evidence-Based Clinical Practice Guidelines in this supplement	Optimal thromboprophylaxis in nonorthopedic surgical patients will consider the risks of VTE and bleeding complications as well as the values and preferences of individual patients
Wood KB [25]	109,609	This is a retrospective cohort study of patients undergoing elective spine surgery in the National Surgical Quality Improvement Program (NSQIP) database and a retrospective cohort analysis at an academic medical center	Pharmacologic prophylaxis, primarily with unfractionated heparin, after elective spine surgery was not associated with a significant reduction in VTE
Yamada K [26]	12484	A systematic review of the English-language literature was undertaken for articles published between January 1993 and December 2008	Exposure and surgery at L4-L5 may be associated with a higher risk of injury than that at L5-S1, though the data are not consistent
Pennington Z [27]	289	Between April 2008 and March 2015, patients with degenerative cervical spine disease, such as compressive myelopathy or radiculopathy, who underwent surgical treatment were prospectively assessed	Female gender and rapidly progressive myelopathy are high-risk factors that predict the development of DVT during the perioperative period of cervical spine surgery
Wang TY [28]	355	A retrospective data set from a comprehensive cancer center was reviewed for adult patients treated for vertebral column tumors	In the present cohort of patients treated for vertebral column tumors, TXA was not associated with increased VTE risk, although high-dose TXA (≥20 mg/kg) was associated with increased odds of DVT or PE
Cloney MB [29]	1346	We evaluated all medical records for 1346 consecutive patients who underwent spinal surgery at Duke University for incidence of DVT within 30 days of surgery and documented all demographic, preoperative, operative, and postoperative variables	Postoperative DVT prophylaxis may be warranted for patients undergoing emergent spine surgery because these patients have significantly higher risk of developing postoperative DVT
Imuro T [30]	6869	The records of 6869 consecutive spine surgeries were retrospectively examined	Anticoagulation reduces the cumulative incidence of VTE after spine surgery. The cumulative incidence of VTEs rises linearly in the first 2 postoperative weeks and then plateaus. Surgeons should consider early initiation of chemoprophylaxis for patients undergoing spine surgery
Cloney MB [31]	6968	Patients with D-dimer levels ≥ 0.5 *μ*g/mL or with a lower extremity manual muscle test (MMT) < grade 3 underwent preoperative US	Preoperative DVT screening by US is advisable for patients with elevated D-dimer levels, lower extremities with MMT < grade 3, or DVT positivity
Zhang H [32]	6869	Examined records from 195 consecutive patients with spinal fractures who underwent spinal stabilization surgeries—among a cohort of 6869 patients who underwent spinal surgery	Compared to all other patients undergoing spine surgery, patients with spinal fractures are more likely to receive chemoprophylactic anticoagulation but have a higher rate of VTE events
Platzer P [33]	2053	Patients who underwent posterior lumbar spinal surgery with internal fixation in the Spine Surgery Center of Peking Union Medical College Hospital (PUMCH) were evaluated	Level of spinal surgery, surgical approach, and motor deficits in the lower extremities were identified as specific risk factors for DVT or PE. Age, sex, obesity, and regular smoking were identified as general risk factors
Purvis TE [34]	6931	The surgical billing database at our institution was queried for inpatients discharged between 2008 and 2015 after the following procedures: atlantoaxial fusion, anterior cervical fusion, posterior cervical fusion, anterior lumbar fusion, posterior lumbar fusion, lateral lumbar fusion	Transfusion using a liberal trigger is associated with increased morbidity, even after controlling for possible confounders. Our results suggest that modification of transfusion practice may be a potential area for improving patient outcomes and reducing costs

The article "Risk Factors for Venous Thrombosis after Spinal Surgery: A Systematic Review and Meta-analysis" was published in 2022. Journal: Comput Math Methods Med.

## Data Availability

The datasets generated during and/or analyzed during the current study are available from the corresponding author on reasonable request.
